# Assessing Compliance to National Guidelines for Pediatric Wrist and Ankle Fractures in a District General Hospital

**DOI:** 10.7759/cureus.19374

**Published:** 2021-11-08

**Authors:** Woo Jae Kim, Jamie Hind, Neil Ashwood

**Affiliations:** 1 Trauma and Orthopedics, Dudley Group NHS Foundation Trust, Dudley, GBR; 2 Trauma and Orthopedics, Oxford University Hospitals NHS Foundation Trust, Oxford, GBR; 3 Trauma and Orthopedics, University Hospitals of Derby and Burton NHS Foundation Trust, Derby, GBR

**Keywords:** pediatric orthopedics, orthopedics surgery, nice guidelines, ankle fractures, wrist fractures

## Abstract

Pediatric ankle and wrist fractures are very common injuries encountered by orthopedic departments. The National Institute of Clinical Excellence has published guidelines that should be adhered to when treating these common fractures. This audit included 560 patients that have sustained wrist and ankle fractures between 2008 and 2019 at Queen Elizabeth Hospital Burton (QHB) that required surgical management. The results show that 99.7% (478/479) wrist fractures and 70.8% (57/81) of ankle fractures received surgical management within the timeframe outlined by NICE. This audit has shown that QHB has been successfully treating wrist fractures within the guidelines set by NICE but has failed to meet the standards for ankle fractures.

## Introduction

The National Institute of Clinical Excellence (NICE) has set guidelines for wrist and ankle fracture management in order to achieve the best functional outcome for patients with less pain and a better range of movement. Distal radius fractures are extremely common injuries in the pediatric population, with one-third of patients suffering this injury before the age of 17 and representing 9% of all childhood injuries [1]. There is evidence that the incidence rates of distal radius fractures are growing [2] and alongside it the rate of surgical intervention [3], resulting in an increased burden on the health service.

Ankle fractures are also common injuries with some literature stating the annual incidence rate to be 1 in 1000 [4] and accounts for 9%-18% of physeal injuries in children aged between 10 and 15 years [5]. There is an ever-growing trend in obesity globally [6], and research has shown there is an increased propensity and severity of ankle injuries in children with a higher body mass index (BMI) [7,8]. NICE has recommended that distal radius fractures should be treated within 72 hours if intra-articular and within seven days if extra-articular, with redisplacement fractures undergoing treatment within 72 hours from when they present. With regard to ankle fractures, they should ideally be treated either on the day of injury or the next day.

As a result of the high prevalence of both wrist and ankle injuries in the pediatric population, it is important to have a set of standards against which treating units can compare their results against. The guidelines produced by NICE provide a framework to which we have been able to compare our results and highlight any discrepancies. The purpose of this retrospective audit was to determine whether Queen Elizabeth Hospital Burton (QHB) has adhered to NICE guidelines when managing pediatric wrist and ankle fractures. This paper not only demonstrates the results of our audit as a tertiary center treating such patients with these injuries but highlights the importance of ongoing assessments of practice.

## Materials and methods

Study design

This was a single-center, retrospective audit carried out in Queens Hospital Burton, a level three trauma unit treating both adult and pediatric populations. This audit collected data for all pediatric patients treated at this unit for an ankle or a wrist injury between 2008 and 2019. During this period, there were 698 patients that were treated in Queens Hospital Burton and were therefore included in our study. These patients were managed with a procedure that included manipulation under anesthesia with or without Kirschner wire (MUA ± K-wire) and open reduction and internal fixation (ORIF).

Inclusion criteria

Strict inclusion criteria were upheld; patients included required an operation secondary to a fracture, and all the data points must be available to be included in the audit.

Exclusion criteria

Patients that did not require operative intervention secondary to a fracture and those with incomplete data sets were excluded from this study. Due to the lack of data, 64 patients were excluded, and a further 74 patients were excluded due to their operative indications not being secondary to a fracture.

Data collection

Data points covered basic patient data of hospital unit number and date of birth as well as the details of the operation including the surgical indication, type of operation, and any complications. The patient’s discharge date and length of stay were also recorded. The data were collected on Microsoft Excel (Microsoft Corporation, New Mexico, USA) and analyzed with basic analysis tools within the program. Current NICE guidelines for the timing of treatment for distal radius and ankle fractures were identified as shown in Table 1.

**Table 1:** NICE guidelines NICE, National Institute of Clinical Excellence.

Timing of surgery for ankle fractures
If treating an ankle fracture with surgery, consider operating on the day of injury or the next day.
Timing of surgery for distal radius fractures
When needed for distal radius fractures, perform surgery within 72 hours of injury for intra-articular fractures and within 7 days of injury for extra-articular fractures. When needed for redisplacement of distal radius fractures, perform surgery within 72 hours of the decision to operate.

## Results

A total of 560 patients were identified and included in the audit; of those, 479 cases consisted of pediatric wrist fractures and the remaining 81 were pediatric ankle fractures (Table 2). Queen’s Hospital Burton has achieved NICE guidance standards with regard to pediatric wrist fracture management with 470 patients (98.1%) having surgical intervention within the 72-hour timeframe (Table 3). Eight patients (1.6%) sustained extra-articular fractures and had received operative intervention within seven days, thus well within the target of NICE guidelines. However, there was one patient (0.3%) who received surgery after >seven days following the redisplacement of his wrist fracture and hence did not receive optimal care.

**Table 2:** Total number of patients

	Total found	Total excluded	Total included
No. of ankles	147	66	81
No. of wrists	551	72	479
Total	698	138	560

**Table 3:** Length of time till operation for wrist fractures

Length of time till operation	Number of wrist operations
Same day	156
Next day	284
Days 2-3	30
Greater than 3 days	8
Greater than 7 days	1

There were 81 pediatric patients who required ankle fixation with 57 (70.4%) of those patients receiving surgical treatment either on the same day or the following day, while 24 patients (29.6%) received operative treatment beyond what has been recommended by NICE guidelines (Table 4). Among the 24 operations that did not meet NICE standards, 17 (70.8%) were children requiring ORIF with the longest time till the operation as seven days.

**Table 4:** Length of time till operation for ankle fractures

Length of time till operation	Number of ankles
Same day	11
Next day	46
2 or more days	24

Complication rates following wrist and ankle surgery were very low; there were six cases (0.012%) where complications arose for wrist fractures with four consisting of failure of fixation, one failure of conservative management following manipulation under anesthesia, and one that resulted in nerve palsy. There was one patient (0.012%) who received ankle surgery that resulted in failure of fixation (Table 5).

**Table 5:** Number of complications

	No. of complications (Wrists)	No. of complications (Ankles)
Total	6	1

## Discussion

The majority of wrist fracture patients received their treatment in a timely manner, with only one wrist fracture patient not being treated within the timeframe recommended by NICE guidelines. This was due to the lack of operating time, which eventually delayed the treatment. This high percentage is perhaps attributed to the fact that a significant proportion of these patients (96.6%) received manipulation under anesthesia with or without Kirschner wire fixation, which is a relatively quick operation.

A recent cohort study of 43 patients found that patients treated with Kirschner wires significantly had shorter operative times than those who were treated with an open reduction and internal fixation (ORIF) procedure [9]. NICE guidelines also give a more lenient timeframe to complete surgical treatment for wrist fractures compared to ankle fractures. The complication rate for wrist fractures was 0.12% (6/479) with four failing following manipulation and cast. A recent meta-analysis that included three randomized controlled trials (RCTs) and three cohort studies reveals that the rate of redisplacement of distal radius fractures following cast immobilization is 45.7%, which is significantly greater than what was found in our audit [10]. A possible explanation for this could be that we achieved anatomic reduction through an image intensifier in the operating room. A recent meta-analysis has been shown to significantly reduce the need for subsequent operative treatment and improve the quality of reduction [11]. Other complications mentioned in the literature following distal radius fractures include non-union, malunion, infections, tendon injuries, and complex pain syndrome, which were not observed in our audit, likely due to the majority of our patients being treated with manipulation under anesthesia with or without Kirschner wires [12].

There was a larger proportion of patients undergoing ankle surgery who did not meet the standards set out by NICE, with 29.6% (24/81) of ankle fractures not receiving appropriate surgical intervention in a timely manner. The standards set by NICE give a short window of opportunity for patients to receive surgical treatment for ankle fractures, primarily due to swelling and soft-tissue complications, which can ensue due to the rubbing of the cast and blistering of the skin [13]. Once there is significant swelling or blistering of the soft tissues, fixation is preferred after the soft tissues have settled. Anatomic reduction is a key with ankle fractures to reduce the risk of chronic pain leading into adulthood, and multiple attempts at reduction should not be performed due to the risk of injury to the physis and growth arrest [14]. One patient was found to have a failure of fixation as a complication. Other complications can include osteochondral defects, malunion, and extensor retinaculum syndrome, which were not found in our audit as they require longer follow-up and further imaging [14,15]. This highlights a limitation in our audit that our problems are confined to more immediate post-operative complications. Further studies could be performed to observe whether there is an increase in the rates of complication if NICE guidelines are not adhered to.

## Conclusions

This audit has shown that QHB has been prioritizing and treating the pediatric patients as per the NICE guidelines for wrist fractures while falling short with regard to ankle fractures. Regardless of this, complication rates for both were very low. Recommendations to improve on this matter are to increase the departmental awareness and education within not only the orthopedic department but also other departments in order to ensure efficient treatment of patients.
